The article "Hidradenitis Suppurativa: A Literature Review Comparing Current Therapeutic Modalities" was published in 2023. Journal: Cureus.

# Hidradenitis Suppurativa: A Literature Review Comparing Current Therapeutic Modalities

**DOI:** 10.7759/cureus.43695

**Published:** 2023-08-18

**Authors:** Urvashi Rathod, Pooja N Prasad, Bhaumikkumar Mukeshbhai Patel, Brinda Patel, Chintankumar Patel, Siddharth Kamal Gandhi, Priyansh Patel

**Affiliations:** 1 Department of Internal Medicine, Narendra Modi Medical College, Ahmedabad, IND; 2 Department of Internal Medicine, Vydehi Institute of Medical Sciences and Research Centre, Bengaluru, IND; 3 Department of Internal Medicine, Shri M. P. Shah Government Medical College, Jamnagar, IND; 4 Department of Internal Medicine, Gujarat Medical Education and Research Society, Sola, Ahmedabad, IND; 5 Department of Internal Medicine, Medical College Baroda, Vadodara, IND

**Keywords:** adalimumab, tnf alpha inhibitors, clindamycin, treatment for hs, hidradenitis suppurativa, hidradenitis suppurativa complication

## Abstract

Hidradenitis suppurativa (HS) is a disease with a poor prognosis, often misinterpreted as an infection, with the highest impact on the patient's quality of life among all the assessed dermatological diseases. The main aim of this study was to compare various therapeutic interventions that are currently available for the treatment of HS. The pathogenesis of HS is not well understood, but it is mostly multifactorial involving a number of factors like genetic factors, androgens, local immunity, microflora, smoking, and obesity. Despite limited evidence on their effectiveness, topical antibiotics and antiseptics are commonly employed. Due to the colonization of bacteria and the presence of biofilms in the sinus tracts formed by HS lesions, systemic antibiotics are commonly employed as the primary form of therapy. In females with HS who experience menstrual flares or display symptoms of polycystic ovary syndrome, hormonal agents are often considered to be a viable and effective therapeutic option. At present, the sole treatment approved by both the Food and Drug Administration and the European Medicines Agency for addressing moderate to severe HS is adalimumab, an antibody that targets tumor necrosis factor alpha. Many surgical procedures in the management of HS aim to address inflammation by eliminating the affected folliculo-pilosebaceous unit, sinus tracts, and associated debris to impede further progression and scarring. HS continues to pose a considerable treatment challenge, necessitating a comprehensive approach for patients. However, the available evidence for most of these treatments is limited, indicating the need for more extensive research to identify the most effective interventions for managing HS.

## Introduction and background

Hidradenitis suppurativa (HS) is a disease, often misinterpreted as an infection, with the high impact on the patient's quality of life among all the assessed dermatological diseases. Globally, it has a prevalence of around 4%, but it is estimated to be around 0.10% in the United States (US) [1]. It is more common in women and is often associated with obesity, smoking, diabetes mellitus, inflammatory bowel disease, and metabolic syndrome [2]. It begins with follicular occlusion in the folliculo-pilosebaceous unit, followed by rupture and an ensuing immune response, where the immune response involves the activation of neutrophilic granulocytes, macrophages, and plasma cells, as well as innate pro-inflammatory cytokines such as interleukins (IL-1β, IL-17), tumor necrosis factor (TNF-α), and interferon (IFN-γ), which leads to a vicious cycle of tissue destruction [3,4]. This painful and deep-rooted condition tends to recur and affects soft tissue in intertriginous regions, such as the axillae, perianal and perineal regions, buttocks, groins, sub-mammary area, and genitals in women [5,6]. These lesions can take various forms, ranging from nodules and abscesses to draining malodorous sinus formation, and can progress to more severe forms such as scarring, open comedones, and fistulas [7].

The article "Hidradenitis Suppurativa: A Literature Review Comparing Current Therapeutic Modalities" was published in 2023. Journal: Cureus.

Treating the patient with HS is the greatest challenge of all time due to its lack of universally accepted standard of care and high rate of recurrence that leads to frustration in both the patients and clinicians. There are diverse treatment strategies aimed at controlling inflammation, scarring, and related comorbidities that include topical and systemic medications, biologics, and surgical interventions. Though the treatment range is wide, not a single approach has proven to be effective in patients with HS [8,9]. Furthermore, the impact on the quality of life of the patients is a very important aspect, and managing the psycho-social aspect is crucial, as the disease is associated with pain, severe discomfort, and embarrassment that causes a profound effect on the patient’s social and mental functioning [10]. In addition to this, the lack of awareness among healthcare professionals can pose a challenge. Many patients are initially misdiagnosed leading to delays in the appropriate treatment and further leading to worsening of the disease [10]. Overall, the challenges in treating the patient with HS need to have a multidisciplinary approach involving dermatologists, surgeons, and various health professionals; however, choosing the right treatment options by comparing them becomes crucial. Therefore, personalized and effective treatment strategies that address the complex nature of HS remain an area of active research. In this review, we compared various therapeutic interventions that are currently available for the treatment of HS.

The article "Hidradenitis Suppurativa: A Literature Review Comparing Current Therapeutic Modalities" was published in 2023. Journal: Cureus.

Methodology

We searched databases like PubMed, Medline, and PubMed Central with keywords including therapeutics, hidradenitis suppurative, microbiology, surgery, drug treatment, and acne inversa. Furthermore, we also included PubMed's medical subject headings (MeSH). We only included studies done on human subjects and published in the English language. Also, we only included studies that were available as free full-text articles. After carefully extracting and analyzing the studies, 36 studies were included in this review.

## Review

Pathophysiology

The pathogenesis of HS is not well understood, but it is mostly multifactorial involving a number of factors such as genetic factors, androgens, local immunity, and microflora [11]. It is also found that tobacco smoking, obesity, and certain mutations can also be related to HS. Nicotine in cigarettes can cause increased neutrophil chemotaxis and production of cytokines (TNF), increased growth of *Staphylococcus aureus*, and decrease in antimicrobial peptides (AMP) such as beta-defensin 11. Obesity is known to be an inflammatory state by itself as adipocytes can increase pro-inflammatory cytokines like TNF and IL-6 that in turn can contribute to the inflammation seen in HS. Also, obesity can cause increased irritation between the skin of the axilla and the groin thus aiding in plugging of the follicles [12]. The role of bacteria in influencing the inflammatory response in HS is debatable, but the elevated levels of S100A7-9, lipocalin-2, and beta-defensins in patients with HS and a good response to treatment with antibiotics have proved that there is a strong association between bacteria and HS. But it is not understood whether the bacteria cause the disease or whether their proliferation in the sinus tracts causes the disease to become severe [13]. In patients with a positive family history of HS, an autosomal dominant mode of inheritance of a mutation in the gamma-secretase complex can be found. These patients tend to have a severe form of HS [12]. Follicular plugging, an increase in the size of the follicular epithelium, and inflammation around the follicles are the main findings in HS. Blockage of the terminal hair follicle can lead to dilatation and the formation of cysts. The inflamed follicle can burst and release the contents that include the hair shaft, keratin fibers, and microbes [14]. The follicular contents released onto the epidermis can trigger other inflammatory pathways like nucleotide-binding oligomerization domain-like receptor protein 3 (NLRP3) inflammasome and toll-like receptor (TLR) signaling thus exacerbating the inflammatory response. Neutrophils, T cells (CD3), B cells (CD19, CD20), plasma cells, natural killer cells (CD56) cells, mast cells, macrophages, and dendritic cells are involved in the inflammatory response [15]. This inflammatory response destroys the structural integrity of the skin leading to the formation of deep-seated sinus tracts. It is seen that the level of matrix metalloproteinase-8 (MMP8 or collagenase 2) is high in patients with HS. MMP8 is an enzyme that helps in breaking down the extracellular components; thus, the elevated level of MMP8 might also be leading to the formation of sinus tracts [16].

The article "Hidradenitis Suppurativa: A Literature Review Comparing Current Therapeutic Modalities" was published in 2023. Journal: Cureus.

Treatment

The prevailing therapeutic approaches primarily revolve around three key elements; first, imparting knowledge and education to patients regarding the condition; second, utilizing medical interventions to address inflammation; and third, employing surgical interventions to manage fistulas, nodules, and scar tissue [17]. The combination of all these factors is essential for controlling the disease. The Hurley classification system is commonly used to categorize HS severity and divides it into three stages as shown in Table 1 [18]. In a cross-sectional study by Huang and Kirchhof, out of all people suffering from HS, 24.4% were at Hurley I, 56.0% were at Hurley II, and 19.5% were at Hurley III [19].

**Table 1:** Hurley classification The information in this table is taken from Horváth et al. [18]. This article is open access and is published under CC-BY-NC licenses.

Stages	Interpretation
Stage I (mild)	Single or multiple abscesses without sinus tracts or scarring
Stage II (moderate)	Recurrent abscesses with sinus tracts and scarring, widely separated lesions
Stage III (severe)	Diffuse skin involvement with multiple interconnected sinus tracts and abscesses

Non-pharmacological Treatment

Counseling patients on preventative measures, such as wearing loose-fitting clothing to minimize friction and promoting weight loss for overweight individuals, can help prevent symptom exacerbation and flare-ups [20]. According to epidemiological research, approximately 90% of individuals with HS are known to smoke cigarettes [21]. Smoking cessation is also critical, as tobacco exposure has been associated with increased HS severity and reduced treatment response [21]. Furthermore, given the increased prevalence of depression and anxiety among HS patients, it is essential to screen for mental health conditions and refer patients to a specialist as needed. It is important to note that while some of these interventions have limited evidence, implementing them in conjunction with medical and surgical therapies may provide a comprehensive approach to HS management [22].

The article "Hidradenitis Suppurativa: A Literature Review Comparing Current Therapeutic Modalities" was published in 2023. Journal: Cureus.

Topical Treatment

Despite limited evidence for their effectiveness, topical antibiotics, and antiseptics are commonly employed [23]. A randomized controlled trial (RCT) with a small sample size revealed that the application of topical clindamycin was effective in reducing nodules, pustules, and abscesses [24]. The use of resorcinol (15%) cream, which has keratolytic, antimicrobial, and anti-inflammatory properties, is also a treatment option for managing HS [25]. Molinelli et al. conducted a study that demonstrated that the use of a resorcinol (15%) cream topically resulted in a notable decrease in both the mean size and quantity of nodules and abscesses, as well as a reduction in pain [26].

Oral Antibiotics

Due to the colonization of bacteria and the presence of biofilms in the tunnels of HS lesions, systemic antibiotics are commonly employed as the primary form of therapy. This approach is favored because of the potential for antibiotics to provide both antimicrobial and anti-inflammatory benefits [5]. For Hurley stages I and II, systemic tetracycline antibiotics are frequently employed as a primary treatment option [27]. A small RCT consisting of 46 patients with mild to moderate HS demonstrated that 500 mg of tetracycline taken twice daily for three months resulted in a reduction in both abscesses and nodules. However, it was found to be comparable in effectiveness to topical clindamycin. Doxycycline, taken at a dosage of 100 mg once or twice daily, is another option for treatment [27]. Based on observational data, a combination therapy consisting of clindamycin (300 mg taken twice daily) and rifampin (300 mg taken twice daily) for a duration of 10-12 weeks has demonstrated efficacy [28]. While antibiotics have been widely utilized and shown to be effective, the emerging evidence of bacterial resistance has restricted their use as a treatment option.

Hormonal Therapies

In females with HS who experience menstrual flares or display symptoms of polycystic ovary syndrome (PCOS), hormonal agents are often considered to be a viable and effective therapeutic option [29]. According to a review of the medical records of 26 female patients who were administered a daily dose of either 100 or 50 mg of spironolactone, the medication was found to be both well-tolerated and efficacious [30].

TNF-Alpha Inhibitors

Currently, the only approved treatment option by both the Food and Drug Administration (FDA) and European Medicines Agency (EMA) for the management of moderate to severe HS is adalimumab (ADA), which is an anti-TNF-α antibody [31]. The use of infliximab (Remicade) has been shown to be effective in reducing pain, improving disease severity, and enhancing the quality of life of patients diagnosed with moderate to severe HS. This medication is administered through intravenous infusion [32].

The article "Hidradenitis Suppurativa: A Literature Review Comparing Current Therapeutic Modalities" was published in 2023. Journal: Cureus.

Miscellaneous

Recent studies have further substantiated the utilization of intralesional steroids for managing flares and localized active lesions in HS [33]. Intralesional corticosteroid therapy is considered a viable approach for isolated HS nodules, believed to operate by activating intralesional glucocorticoid receptors and subsequently inhibiting the production of proinflammatory cytokines. The use of intralesional injections of glucocorticoids has also demonstrated encouraging outcomes. Notably, triamcinolone, when administered for individual lesions, has proven effective at concentrations ranging from 2 to 5 mg/ml [34].

Surgical Treatment

Surgical procedures in the management of HS aim to address inflammation by eliminating the affected folliculo-pilosebaceous unit, sinus tracts, and associated debris to impede further progression and scarring [35]. Local techniques employed include punch debridement, unroofing/deroofing, skin-tissue-sparing excision with electrosurgical peeling, and laser excision [35]. Table 2 shows different therapeutic modalities and their effectiveness.

**Table 2:** Therapeutic modalities for HS HS: hidradenitis suppurativa

Treatment/management option	Mechanism of action	Pros	Cons
Lifestyle modifications [20-22]	Weight management to reduce pressure on affected areas. Wearing loose-fitting clothing to minimizes friction and irritation. Smoking cessation to reduce disease severity and progression.	Complementary to medical treatments, can help reduce flare-ups and improve the overall well-being, no associated side effects.	May not be sufficient as a standalone treatment; requires commitment and lifestyle changes.
Topical medications [23-26]	Antibacterial washes/soaps to reduce bacterial colonization and prevent infection. Topical antibiotics (e.g., clindamycin, erythromycin) to target local infections and reduce inflammation. Retinoids (e.g., tretinoin) to prevent blockage of hair follicles and reduce inflammation.	Easy to use and apply, may provide relief for mild cases or early stages of HS, few systemic side effects.	Limited efficacy in moderate to severe cases; may not fully eliminate symptoms. Some individuals may experience skin irritation or dryness.
Systemic antibiotics [5,27,28]	Antibiotics such as tetracyclines (e.g., doxycycline) or rifampicin to target bacterial overgrowth and reduce inflammation.	Effective in controlling infection and reducing inflammation, may provide long-term remission in some individuals, can be combined with other treatments for better outcomes.	May require prolonged courses of antibiotics; potential for antibiotic resistance; possible systemic side effects (e.g., gastrointestinal disturbances, photosensitivity).
Intralesional injections [33,34]	Corticosteroids (e.g., triamcinolone) injected directly into individual lesions to reduce inflammation and promote healing.	Effective in reducing pain, and inflammation, and promoting healing in localized lesions; can be used for acute flares or individual persistent lesions.	Only suitable for localized lesions; may cause temporary skin atrophy or hypopigmentation at the injection site. Limited long-term efficacy.
Systemic immunosuppressive therapy [31,32]	Oral retinoids (e.g., isotretinoin) to normalize keratinization and reduce inflammation. Biologic agents (e.g., adalimumab, infliximab) to target specific inflammatory pathways.	Can be effective in severe cases or those resistant to other treatments; may provide long-term remission. Biologic agents have shown promising results in clinical trials. Isotretinoin can address acne-like symptoms associated with HS.	Requires close monitoring and regular blood tests; potential for systemic side effects and interactions. Biologic agents can be expensive and may increase the risk of infections. Isotretinoin has teratogenic effects and requires contraception.
Surgical interventions [35]	Incision and drainage to relieve pain and remove pus from abscesses. Wide excision for surgical removal of affected skin and tissue. Laser therapy for ablation of affected tissue and hair follicles.	Can provide temporary or long-term relief in severe cases; may be necessary for recurrent or persistent abscesses. Laser therapy may help reduce hair follicle blockage.	Surgical interventions carry risks, such as infection, scarring, or wound-healing complications; may require multiple procedures. Lesions may recur after surgery.

Limitations

This study has some limitations, one of which is the absence of sufficient high-level evidence, such as meta-analyses. All the identified studies were based on a limited number of observational studies, case reports, case series, systematic reviews, and animal studies available. These studies exhibited heterogeneity in the sample size and measurement of variables. Furthermore, not all the studies assessed had similar variables and secondary outcomes. Also, this review only included papers written in the English language. In addition, more research is required to establish effective first-line treatment for HS.

The article "Hidradenitis Suppurativa: A Literature Review Comparing Current Therapeutic Modalities" was published in 2023. Journal: Cureus.

## Conclusions

In this review, we compared various therapeutic interventions that are currently available for the treatment of HS. Furthermore, we discussed less well-elucidated pathogenesis of HS and multifactorial involving factors such as androgens, local immunity, microflora, obesity, tobacco smoking, and so forth. Due to the complex nature of HS, patients may require one or more adjuvant therapies to manage associated infections, flare-ups, obesity, smoking cessation, and psychological impacts. Numerous medical treatments are available for HS such as local and systematic antibiotics, retinoids, antiandrogens, immunosuppressive therapies, anti-inflammatory agents, and radiotherapy. A number of local surgical techniques have also been proven beneficial such as punch debridement, unroofing/deroofing, skin-tissue sparing excision with electrosurgical peeling, and laser excision. Currently, the only FDA-approved biological drug for the management of severe HS is adalimumab, which acts as a TNF-α blocker. While some cytokine selective inhibitors are under early stages of development and research, they have not yet received approval. As a result, HS remains a complex condition to treat, often requiring a combination of approaches. However, the available evidence for most of these treatments is limited, highlighting the necessity for additional randomized controlled trials in the future to determine the most effective interventions for HS management.
